# Stent Migration Following Endovascular Intervention in May-Thurner Syndrome

**DOI:** 10.7759/cureus.29714

**Published:** 2022-09-28

**Authors:** Dominick Steck, Suresh Keshavamurthy, Akshay Kumar, Sean Lyden, Eric Roselli

**Affiliations:** 1 Surgery, University of Washington School of Medicine, Seattle, USA; 2 Cardiothoracic Surgery, University of Kentucky, Lexington, USA; 3 Cardiothoracic Surgery, Cleveland Clinic Foundation, Cleveland, USA; 4 Vascular Surgery, Cleveland Clinic Foundation, Cleveland, USA

**Keywords:** right ventricle, right atrium, common iliac vein, may-thurner syndrome, stent migration, tricuspid regurgitation, tricuspid valve, foreign body

## Abstract

Developments in endovascular therapies have made stenting a common practice in the treatment of peripheral vascular diseases, including venous disorders such as May-Thurner syndrome. The placement of a stent in the venous system carries the risk of stent migration which although small occurs with a 3% incidence rate and can be life-threatening given the risk of pulmonary infarction, tricuspid regurgitation, and right-sided heart failure. Herein we report a case of stent embolization from the common iliac vein into the right side of the heart causing tricuspid regurgitation. After the failure of percutaneous approach to retrieve the stent, it was successfully removed using a minimally invasive right thoracotomy approach along with repair of the tricuspid valve.

## Introduction

The use of endovascular techniques for the treatment of both venous and arterial systems has become an integral part of our armamentarium. A possible complication of these endovascular interventions, which occurs occasionally (up to 3% incidence rate), is incorrect placement of a stent or the migration of a stent after its deployment. These can be hazardous and potentially life-threatening events owing to secondary vascular complications. Correction or removal of an embolized or malpositioned stent is required to manage these complications [1]. In addition to the danger of thrombosis, permanent vessel wall trauma perforations are serious sequelae; other complications include distal embolization of arterial stents and central embolization of venous stents. The latter is associated with cardiac complications including arrhythmias, injury of the valves or papillary muscles, or possible arterial occlusion in the case of pulmonary artery embolization. If the patient has a patent foramen ovale the migrated stent might even cause neurovascular complications. While endovascular techniques are available to retrieve the vagabond stent, surgical extraction continues to be the alternative.

## Case presentation

A 30-year-old male initially presented to the emergency department of an outside hospital when he suddenly experienced chest pain as a severe pressure-like sensation located in the mid-sternal region. His past medical history included varicose veins and leg pain, and he underwent multiple saphenous ablations which brought relief for only a short period of time. He was recently diagnosed with May-Thurner syndrome, when a narrowing of the distal part of the left iliac vein was detected, and the vessel was stented (14x80 mm Zilver(R) stent) just four months before the current presentation. The patient reported that the pain got worse when in a supine position and with deep inspiration, and improved when sitting up. He also complained of minimal shortness of breath, but denied any other symptoms. An acute coronary syndrome was ruled out [creatine kinase (CK) was elevated but the other cardiac biomarkers were negative], the EKG did not show any significant changes, and the X-ray chest was normal (Figure 1).

**Figure 1:** X-ray Chest showing mild congestion

The patient was subsequently discharged home with pain medication (hydrocodone/paracetamol). While at home the pain continued to worsen, his primary care physician repeated EKG which revealed sinus tachycardia with diffuse ST elevations with reciprocal ST depression in aVR; PR segment elevation in aVR; PR segment depression in V1. His 2D echocardiography showed a 3.7 x 1.8 cm echodensity in the right ventricle [right iliac stent that migrated to the right ventricle (Figure 2)] and severe tricuspid regurgitation (Figure 3).

**Figure 2:** 2D Transthoracic echocardiography parasternal short axis view showing 3.7 cm x 1.8 cm echodensity in the right ventricle.

**Figure 3:** Continuous Wave Doppler imaging on transthoracic echocardiography (TTE) showing severe tricuspid regurgitation.

A large part of the stent was lying within the right ventricle (Video 1) and a small part was enmeshed in the tricuspid valve apparatus leading to severe regurgitation (Video 2).

**Video 1:** 2D Transthoracic echocardiography short axis showing stent within the right ventricle and circumferential pericardial effusion

**Video 2:** 2D Transthoracic echocardiography short axis view at the mid ventricle level demonstrating the stent in the right ventricle abutting the tricuspid valve with severe tricuspid regurgitation

The patient underwent a cardiac catheterization which showed normal coronary arteries but noted a foreign body in the right ventricle. His chest pain improved somewhat with the IV morphine therapy. The following day the patient was transferred to our institution for further management. A percutaneous approach to retrieve the stent from the right heart was initially attempted. Transesophageal echocardiography showed severe (4+) tricuspid regurgitation, moderate pericardial effusion, and the patent foramen ovale (PFO). An attempt was made to retrieve the stent via the right internal jugular vein approach; however, it fractured during this procedure and only a small fragment of the stent could be removed. At this point, it became clear that it would be very difficult to remove the stent through percutaneous access, and therefore an open surgical approach was adopted.

Since we already had access to the superior vena cava, it was decided to take advantage of that and use it for venous drainage for cardiopulmonary bypass. A right thoracotomy was chosen instead of a full sternotomy as a less invasive approach and to allow a quick recovery during the postoperative course. The patient underwent bicaval cannulation, 18F SVC, 20F IVC and a Left Femoral arterial 20F cannula after systemic heparinization. Caval snares were tightened. Upon opening the right atrium a PFO (patent foramen ovale) was found and closed with a running stitch. The largest part of the stent was trapped between the anterior and septal leaflets of the tricuspid valve, in addition, there was a mass and vegetation underneath this area on the ventricular side of the tricuspid valve, and the valve showed signs of acute inflammation. Multiple segments of the partially fragmented stent were carefully removed. After we were sure that all parts of the stent were removed the heart was irrigated copiously. The stent had caused multiple small perforations in the tricuspid valve, these were repaired with 5-0 ethibond sutures. A commissuroplasty in the region between the anterior and the septal leaflet bicuspidization procedure using a Kay technique [2] was performed. The right atrium was then closed. The patient was subsequently weaned from bypass, fluoroscopy and the transesophageal echocardiogram (TEE) showed no further evidence of foreign body in the heart, there was residual 3+ tricuspid regurgitation with a mean gradient of 3 mm Hg, but significantly better compared to the preoperative situation. After decannulation and heparin reversal, a chest tube was placed in the right pleural space. The patient was taken to the ICU in a stable condition.

Immediately after waking up from the general anesthesia, the patient felt significantly better. The chest X-ray on the second postoperative day revealed small bilateral pleural effusions which were treated with diuretics. On the fourth postoperative day an echocardiogram was performed which showed 3+ tricuspid regurgitation. He was started on vancomycin, however, his cultures finally came as negative. On the sixth postoperative day, the patient was discharged home. The clopidogrel therapy that the patient was on before the incident was stopped and he was put on acetylsalicylic acid.

## Discussion

Although percutaneous endovascular stenting has emerged as the primary treatment option for symptomatic venous outflow obstruction during the past decade, stent migration remains a recognized complication with significant morbidity and mortality. Recent studies suggest that migration is more likely to occur with shorter length (60 mm) and smaller diameter (14 mm) stents, with the combination the most common. Stents should be of the appropriate size in both length and diameter for the intended vascular bed. This issue might be related to inadequate oversizing of the stent, inaccurate positioning of the stent within the lesion, or inaccurate vessel measurement. The iliocaval segment was found to have the highest incidence of migration, followed by the central and renal vein stents.

May-Thurner syndrome is named after Robert May and Josef Thurner who published the results of their research on thromboses of the left pelvis veins in 1957. The right common iliac crosses the left iliac vein causing compression of the vein with an ensuing permanent irritation of the vessel that leads to endothelial proliferation with a resulting formation of the spur. The spur causes stenosis of the lumen that impedes the blood flow and causes the emergence of thrombosis [1].

Kibbe et al. conducted a radiologic study on the degree of compression of the iliac veins at the site of the crossing of the right common iliac artery in patients that had no history of thrombotic incidences in this region. Twenty-four percent of all patients had greater than 50% compression; 66% of all patients had at least 25% compression of the left iliac vein. This led to the assumption that a certain degree of compression of the left iliac vein may be normal and does not result in an increased risk for the development of thrombosis in this region [3].

Regardless of the mentioned findings, endovascular treatment in the form of stenting is a well-established therapy for patients with May-Thurner syndrome and thrombosis of the lower extremity [4]. Several studies on the long-term outcome of this treatment have been conducted. Kim et al. analyzed the data of 21 patients with deep vein thrombosis (16 acute iliofemoral venous thromboses, five with chronic venous outflow obstruction with thrombus) that had been diagnosed with May-Thurner syndrome during the diagnostic workup. Eighteen of these 21 patients underwent balloon angioplasty and placement of a wall stent, and three patients underwent balloon angioplasty alone. Follow-up on all three angioplasty-only patients three to six months later showed restenosis and thrombosis, whereas the follow-up (in 17 of the 18 patients) six months after the stent implantation showed thrombus formation in only two of the 17 patients [5]. Titus et al. performed lower extremity venous stenting in 36 patients, out of which 15 had been diagnosed with May-Thurner syndrome, the 24 months patency rate was 100% [6].

Literature review, regarding foreign bodies in the right heart, showed that there have been several reports of cases of cava filters ending up in the right heart, with fatal consequences at times. Nicholson et al. conducted a retrospective study in which they evaluated 80 patients who had received either a Bard Recovery or Bard G2 filter. In five patients of the Bard Recovery group (28 patients) one or more fragments were embolized to the heart. Three of these patients experienced ventricular tachycardia and/or tamponade, out of the three patients one died [7].

In our patient, a Zilver(R) nitinol stent was used. It consists of a structure of interconnected Z-shaped cells. Taneja and Rajan reported on a case of a patient who had undergone a liver transplant and 20 months later suffered from stenosis of the inferior vena cava, therefore two Zilver(R) stents were deployed in this vessel. One month later a CT scan showed that the stents had migrated en bloc into the right ventricle. A percutaneous approach to retrieve the stents was initiated, simultaneously with two snares through both the femoral vein and the internal jugular vein, to be able to pull on and distend the two big stents. During this maneuver, the stents fractured, but it was possible to recover the fragments through multiple snaring maneuvers [8].

The embolization of a stent placed for the treatment of May-Thurner syndrome seems to be very rare though. Mullens et al., however, have reported a case of a 55-year-old woman who had undergone placement of two stents in the left iliac vein. The patient presented with dyspnea and fatigue and TEE showed that both stents had embolized to the right heart. One was found in the ventricular outflow tract, the other attached to the tricuspid valve causing severe regurgitation. The stents had to be removed surgically and the tricuspid valve repaired, by the addition of neochordae in addition to ring annuloplasty [9]. We didn’t want to leave behind an implant in order to avoid the risk of endocarditis and therefore performed a Kay repair [2] which was also expeditious. In retrospect we could have used a rigid annuloplasty ring which has been shown to provide early and sustained reduction of tricuspid regurgitation [10].

## Conclusions

Stent migration from the venous system into the right side of the heart can be catastrophic resulting from acute right ventricular outflow tract obstruction. Endovascular approach to retrieve the migrated stent should be utilized whenever feasible. In cases where it is not successful and there is severe damage to other heart structures including valves, the open approach is necessitated to remove the stent, repair the valve and address comorbid issues.

## References

[1] May R, Thurner J (1957). The cause of the predominantly sinistral occurrence of thrombosis of the pelvic veins. Angiology.

[2] Kay JH (1992). Surgical treatment of tricuspid regurgitation. Ann Thorac Surg.

[3] Kibbe MR, Ujiki M, Goodwin AL, Eskandari M, Yao J, Matsumura J (2004). Iliac vein compression in an asymptomatic patient population. J Vasc Surg.

[4] De Bast Y, Dahin L (2009). May-Thurner syndrome will be completed?. Thromb Res.

[5] Kim JY, Choi D, Guk Ko Y, Park S, Jang Y, Lee do Y (2006). Percutaneous treatment of deep vein thrombosis in May-Thurner syndrome. Cardiovasc Intervent Radiol.

[6] Titus JM, Moise MA, Bena J, Lyden SP, Clair DG (2011). Iliofemoral stenting for venous occlusive disease. J Vasc Surg.

[7] Nicholson W, Nicholson WJ, Tolerico P (2010). Prevalence of fracture and fragment embolization of Bard retrievable vena cava filters and clinical implications including cardiac perforation and tamponade. Arch Intern Med.

[8] Taneja M, Rajan DK (2006). Percutaneous removal of migrated nitinol stents from the right ventricle. J Vasc Interv Radiol.

[9] Mullens W, De Keyser J, Van Dorpe A, Meuris B, Flameng W, Herregods MC, Van de Werf F (2006). Migration of two venous stents into the right ventricle in a patient with May-Thurner syndrome. Int J Cardiol.

[10] Navia JL, Nowicki ER, Blackstone EH (2010). Surgical management of secondary tricuspid valve regurgitation: annulus, commissure, or leaflet procedure?. J Thorac Cardiovasc Surg.

